The article "Famous Faces Demand Attention Due to Reduced Inhibitory Processing" was published in 2011. Journal: PLoS One.

# Famous Faces Demand Attention Due to Reduced Inhibitory Processing

**DOI:** 10.1371/journal.pone.0020544

**Published:** 2011-05-31

**Authors:** Liana Machado, Hayley Guiney, Andrew Mitchell

**Affiliations:** Department of Psychology and Brain Health Research Centre, University of Otago, Dunedin, New Zealand; Macquarie University, Australia

## Abstract

People have particular difficulty ignoring distractors that depict faces. This phenomenon has been attributed to the high level of biological significance that faces carry. The current study aimed to elucidate the mechanism by which faces gain processing priority. We used a focused attention paradigm that tracks the influence of a distractor over time and provides a measure of inhibitory processing. Upright famous faces served as test stimuli and inverted versions of the faces as well as upright non-face objects served as control stimuli. The results revealed that although all of the stimuli elicited similar levels of distraction, only inverted distractor faces and non-face objects elicited inhibitory effects. The lack of inhibitory effects for upright famous faces provides novel evidence that reduced inhibitory processing underlies the mandatory nature of face processing.

## Introduction

Faces fall into a special class of stimuli that demands processing under circumstances in which other types of distractors can be ignored [1], [2]. The attentionally demanding nature of faces has been demonstrated even when the faces never appear in task relevant positions [3], [4]. Prioritized processing of faces can afford obvious evolutionary advantages due to their high level of biological significance. The current research investigated the mechanism underlying this prioritized processing. Previous studies suggest that faces receive enhanced processing, thereby rendering faces more difficult to ignore than non-face stimuli [2]. Enhanced excitatory processing specific to faces could fully account for the difficulty ignoring faces. Alternatively, considering the importance of inhibitory processing during selective attention [5], [6], it could be the case that a lesser amount of inhibitory processing specific to distractors that depict faces contributes to this phenomenon.

To address the possibility that reduced inhibition underlies the mandatory nature of face processing, we utilized a focused attention paradigm that tracks the influence of a distractor over time and provides a measure of inhibitory processing [6], [7]. During each trial, a peripheral distractor appears prior to a central target, and the influence of the distractor on responses to the target are measured (see Figure 1). Our previous research using this paradigm and non-face stimuli established that distractors initially facilitate related processing, as evidenced by faster response times when the subsequent target matches the distractor compared to when the distractor and target are incompatible, which produces a positive compatibility effect. However, after a few hundred milliseconds, mounting inhibition of the distracting information delays responses to related stimuli, as evidenced by slower response times when the subsequent target matches the distractor compared to when the distractor and target are incompatible, which produces a negative compatibility effect. The magnitude of the negative compatibility effect indicates the extent to which the distractor was inhibited.

The article "Famous Faces Demand Attention Due to Reduced Inhibitory Processing" was published in 2011. Journal: PLoS One.

**Figure 1:** Trial sequence. A distractor appeared above or below fixation at random and was either the same as (compatible) or different than (incompatible) a subsequent central target. The distractor and the target were both either upright or inverted, depending on the version. Participants identified the central target on all trials by pressing one of two buttons.

By considering the time course of distraction, we aimed to expose the processing fate of distractors that depict faces during focused, selective attention. We used famous faces because they have been shown to be especially demanding of attention [8]–[10]. Inverted versions of the faces served as control stimuli, providing equivalent visual properties while disrupting face processing [11], [12]. Prior to assessing the effects of face stimuli, we confirmed that the biphasic pattern of effects reported by Machado et al. [6], [7] extends to complex stimuli by using images of non-face objects as the stimuli. If reduced inhibitory processing underlies the difficulty people exhibit ignoring faces, then distractors depicting upright faces should be subjected to less inhibition during selective attention, relative to inverted faces and non-face stimuli. In the context of the current paradigm, this should result in an attenuated negative compatibility effect specific to upright faces.

## Methods

### Ethics Statement

This research was approved by the University of Otago Human Ethics Committee, and all participants provided written informed consent prior to participation.

### Participants

Ninety young adults recruited at the University of Otago participated either in exchange for NZ$12.50 or in association with a course. Thirty completed the version with non-face objects (mean age = 22, SD = 5, range = 18–42; 14 males; 27 right handed), thirty completed the version with upright faces (mean age = 21, SD = 2, range = 18–27; 15 males; 26 right handed) and thirty completed the version with inverted faces (mean age = 21, SD = 3, range = 18–31; 10 males; 24 right handed). All participants reported no previous neurological history and normal or corrected-to-normal vision.

The article "Famous Faces Demand Attention Due to Reduced Inhibitory Processing" was published in 2011. Journal: PLoS One.

### Stimuli and procedure

All stimuli appeared on a white background. For the version with non-face objects, two grey-scale images, one of a butterfly and the other of a wheel, served as the target and distractor stimuli. Each non-face object subtended 1° both vertically and horizontally, and 2° separated the target and distractor (edge to edge). For the versions with face stimuli, two grey-scale images portraying faces of famous people (George Clooney—actor and Helen Clark—New Zealand Prime Minister) served as the target and distractor stimuli. Each face subtended 3° vertically and 2.4° horizontally, and 2.5° separated the target and distractor (edge to edge). Relative to the non-face objects, the size of the face stimuli had to be increased because pilot testing showed that 1° faces did not elicit any compatibility effects (i.e., the distractors were entirely ineffective). In the versions with non-face objects and upright faces, both the distractor and the target always appeared right-side up. In the version with inverted faces, both the distractor and the target always appeared upside down. In all versions, the two images were each assigned to one of the two buttons on a DirectN Response Box (Empirisoft, New York), with the stimulus-response mapping counterbalanced across participants.

At the start of each trial (see Figure 1), a black fixation dot with a diameter extending .3° of visual angle appeared at the center of the screen. After 500 ms elapsed, one of the images appeared either above or below the fixation dot. This initial image served as the distractor. After a variable interval (50, 350, 650, or 950 ms), another image appeared at the center of the screen (occluding the fixation dot). This central image served as the target. The distractor was either the same as the target (compatible) or different than the target (incompatible). The distractor was positioned above or below the target in order to prevent spatial compatibility effects based on the side of the distractor and the side of the response [13], [14]. The position of the distractor (above or below), the distractor-target onset asynchrony (50, 350, 650 or 950 ms), the distractor identity, and the target identity were randomly selected before each trial with the constraint that each occurred equally often and all conditions were counterbalanced within each block of 32 trials. The code for the experiment relied on MATLAB (The MathWorks, Natick, MA) and The Psychophysics Toolbox [15], [16].

The article "Famous Faces Demand Attention Due to Reduced Inhibitory Processing" was published in 2011. Journal: PLoS One.

Participants sat 57 cm from the screen in a dimly lit room. At the start of the experiment, the computer displayed the stimulus-response mapping. The experimenter instructed participants to fixate on the center of the screen throughout the experiment and, when a stimulus appeared at center, to press the assigned button as quickly as they accurately could using the index and middle fingers of their dominant hand. Note that the experimenter never referred to the identities of the images. The trial ended when the computer recorded either a correct response or an error, at which time the distractor and target disappeared, leaving the screen blank for 2000 ms before the next trial started. An error tone sounded if the participant depressed the wrong button, responded within 100 ms after target onset, or failed to respond within 2000 ms after target onset. All participants completed 32 practice trials followed by 320 test trials, which were divided into 10 blocks. Between blocks, the stimulus-response mapping display reappeared and participants were given the opportunity to rest. For the versions with face stimuli, after completing the experiment, participants were shown the faces in the upright orientation and asked whether they recognized them. Correct identification of the two faces was an inclusion criterion; ten additional participants did not meet this criterion and were excluded.

## Results

An analysis of variance (ANOVA) was conducted on the median reaction times (RTs) of the correct responses and the error rates with distractor-target SOA (50, 350, 650, or 950 ms) and distractor-target compatibility as within-subjects factors. Table 1 and Figure 2 summarize the data for non-face objects, upright faces, and inverted faces.

**Figure 2:** For each version (non-face objects, upright faces, and inverted faces), the size of the compatibility effect in milliseconds for each distractor-target SOA. The compatibility effect equals response latencies on incompatible trials minus response latencies on compatible trials.

**Table 1:** Mean (*M*) and Standard Deviation (*SD*) of the Median Reaction Times (in ms) and Error Rates (*%E*) for Each Condition.

		SOA											
		50			350			650			950		
Version	Condition	*M*	*SD*	*%E*	*M*	*SD*	*%E*	*M*	*SD*	*%E*	*M*	*SD*	*%E*
Non-face objects	Incompatible	529	65	2.3	477	64	2.8	449	61	2.3	439	73	2.7
	Compatible	506	69	2.0	461	66	1.5	461	71	2.5	453	67	2.4
	**Effect**	**23**			**16**			**−12**			**−14**		
Upright faces	Incompatible	529	64	2.8	497	67	2.0	483	68	2.1	476	64	1.8
	Compatible	506	67	1.8	469	71	2.0	479	71	2.3	475	70	1.7
	**Effect**	**23**			**28**			**4**			**1**		
Inverted faces	Incompatible	546	76	3.3	500	75	2.5	480	69	2.1	473	71	1.3
	Compatible	523	77	2.3	480	71	3.0	483	66	2.0	486	67	3.0
	**Effect**	**23**			**20**			**−3**			**−13**		

*Note*. For each stimulus onset asynchrony (SOA), the compatibility effect (i.e., incompatible minus compatible) appears in boldface.

The article "Famous Faces Demand Attention Due to Reduced Inhibitory Processing" was published in 2011. Journal: PLoS One.

### Non-face Objects

#### Reaction times

Distractor-target SOA produced a main effect, *F*(3, 87) = 80.791, *p*<.001, which reflected a quickening of RTs as the interval between distractor and target onset increased. There was no main effect of compatibility (*p*>.5), but SOA and compatibility did interact, *F*(3, 87) = 13.855, *p*<.001, indicating that the compatibility effect depended on the interval between distractor and target onset. To investigate this interaction, we compared RTs on compatible versus incompatible trials for each SOA. The results revealed faster RTs on compatible than incompatible trials when the distractor preceded the target by 50 ms, *t*(29) = 5.849, *p*<.001, or 350 ms, *t*(29) = 2.368, *p* = .023. In contrast, for the 650 ms SOA, RTs had a tendency to be slower on compatible than incompatible trials, *t*(29) = 1.747, *p* = .088. For the 950 ms SOA, RTs were significantly slower on compatible than incompatible trials, *t*(29) = 2.254, *p* = .030.

#### Errors

Errors occurred on 2.3% of the trials. The ANOVA yielded neither significant effects nor an interaction (*p*>.2 in all cases).

### Upright Faces

#### Reaction times

Distractor-target SOA produced a main effect, *F*(3, 87) = 33.404, *p*<.001, which reflected a quickening of RTs as the interval between distractor and target onset increased. Compatibility also produced a main effect, *F*(1, 29) = 13.528, *p* = .001, indicating faster RTs on compatible versus incompatible trials. SOA and compatibility interacted, *F*(3, 87) = 8.126, *p*<.001, showing that the compatibility effect depended on the interval between distractor and target onset. To investigate this interaction, we compared RTs on compatible versus incompatible trials for each SOA. The results revealed faster RTs on compatible than incompatible trials when the distractor preceded the target by 50 ms, *t*(29) = 4.995, *p*<.001, or 350 ms, *t*(29) = 4.551, *p*<.001. For the 650 and 950 ms SOAs, RTs did not depend on compatibility (*p*>.5).

#### Errors

Errors occurred on 2.1% of the trials. The ANOVA yielded neither significant effects nor an interaction (*p*>.3 in all cases).

### Inverted Faces

#### Reaction times

The ANOVA revealed a main effect of SOA, *F*(3, 87) = 63.043, *p*<.001, which reflected the quickening of RTs as the SOA increased. Compatibility did not produce a main effect (*p*>.05); however, it did interact with SOA, *F*(3, 87) = 11.115, *p*<.001. We investigated this interaction by comparing compatible and incompatible trials for each SOA. Consistent with the data for upright faces, the results revealed faster RTs on compatible than incompatible trials when the distractor preceded the target by 50 ms, *t*(29) = 5.239, *p*<.001, or 350 ms, *t*(29) = 3.019, *p* = .005. For the 650 ms SOA, RTs did not depend on compatibility (*p*>.6). Contrary to the data for upright faces, RTs were slower on compatible than incompatible trials at the 950 ms SOA, *t*(29) = 2.110, *p* = .041. This pattern of compatibility effects replicates that reported previously for non-face stimuli [6], [7].

The article "Famous Faces Demand Attention Due to Reduced Inhibitory Processing" was published in 2011. Journal: PLoS One.

#### Errors

Errors occurred on 2.4% of the trials. The ANOVA showed no main effects (*p*>.2 in all cases); however, distractor-target SOA and compatibility interacted, *F*(3, 87) = 3.652, *p* = .015. A separate analysis of the compatibility effects at each SOA revealed more errors on compatible than incompatible trials when the distractor preceded the target by 950 ms, *t*(29) = 2.911, *p* = .007. Thus, consistent with the RT data, at the long distractor-target SOA accuracy suffered when the target matched the distractor. For the 50, 350 and 650 ms SOAs, the frequency of errors did not depend on compatibility (*p*>.1).

### Upright Faces versus Inverted Faces

#### Reaction times

A between-subjects comparison of the versions with upright versus inverted faces showed no significant influences of face orientation (*p*>.06 in all cases). Planned analyses of the RT data for upright versus inverted faces at each SOA revealed a trend for a difference in the effect of compatibility at the 950 ms SOA, *F*(1, 58) = 2.857, *p* = .093, which reflects the occurrence of a significant negative compatibility effect for inverted but not upright faces. The effect of compatibility did not depend on face orientation at the 50, 350 or 650 ms SOAs (*p*>.5 in all cases).

#### Errors

A between-subjects comparison of the versions with upright versus inverted faces showed no significant influences of face orientation (*p*>.1 in all cases). Planned analyses of the error rates for upright versus inverted faces at each SOA revealed a significant difference in the effect of compatibility at the 950 ms SOA, *F*(1, 58) = 5.800, *p* = .018, which reflects the occurrence of a significant negative compatibility effect for inverted but not upright faces. The effect of compatibility did not depend on face orientation at the 50, 350 or 650 ms SOAs (*p*>.5 in all cases).

## Discussion

In an effort to determine whether reduced inhibitory processing underlies the mandatory nature of face processing, we assessed the time course of distraction for upright and inverted famous faces, as well as for non-face objects. We predicted that weaker inhibitory processing may occur when the distractor engages face processing (upright faces), relative to when the distractor does not engage face processing (inverted faces and non-face objects). On all trials, the target appeared at center after the onset of a peripheral distractor. The interval between distractor onset and target onset varied, so that the influence of the distractor could be tracked over time. Distractor-target compatibility effects served as indicators of distractor processing, with positive compatibility effects reflecting excitatory distractor processing and negative compatibility effects reflecting inhibitory distractor processing.

The article "Famous Faces Demand Attention Due to Reduced Inhibitory Processing" was published in 2011. Journal: PLoS One.

The results show that while all of the stimuli elicited equivalent distraction initially, only non-face objects and inverted faces elicited a negative compatibility effect at longer distractor-target delays, as evidenced by increased error rates and delayed response latencies when the target matched the distractor. This indicates that a buildup of distractor inhibition hindered responses for non-face objects and inverted faces only. The biphasic pattern of compatibility effects for non-face objects and inverted faces replicates that shown previously for simple non-face stimuli (red and green squares) [6], [7]. For upright faces, the compatibility effect reduced as the distractor-target SOA lengthened, which suggests that some inhibitory processing of upright distractor faces may have occurred. However, in contrast to the effects for non-face objects and inverted faces, the compatibility effect did not reverse into a negative compatibility effect for upright faces, which indicates that distractors that depicted upright faces were subjected to less inhibitory processing. This indication that reduced inhibitory processing occurred for upright distractor faces was bolstered by a between-version difference in the compatibility effect at the long SOA for upright versus inverted faces. These results provide novel evidence that reduced inhibitory processing underlies prioritized processing of famous faces. In addition to furthering our understanding of face processing, the current results provide key insight for the interpretation of numerous recent studies reporting on general mechanisms of selective attention that used face stimuli as distractors [17]–[19].

### Face processing

The extent to which faces demand attention over and above other classes of objects has attracted considerable interest over recent years [2]. Previous research attributed this phenomenon to enhanced processing specific to faces; however, the potential role of inhibition in this prioritized processing has remained largely uninvestigated until now. Our data clearly demonstrate that less inhibition was used when the distractor engaged face processing (upright distractor face) compared to when the distractor face was inverted, thereby disrupting face processing. For upright faces, although the amount of distractor inhibition was insufficient for the compatibility effect to reverse at the long SOA, the fact that the compatibility effect weakened as the SOA increased converges with previous reports that attention can modulate the neural response to face stimuli [20], [21] and also that the attentional bias toward faces is subject to voluntary control [22]. Note, however, that our face stimuli included hair and hence the attenuation of the compatibility effect as the SOA increased may reflect inhibitory processing of non-facial features.

The article "Famous Faces Demand Attention Due to Reduced Inhibitory Processing" was published in 2011. Journal: PLoS One.

Superficially, the lack of a negative compatibility effect for upright faces seems inconsistent with a previous report of an inhibitory effect for face distractors [23]. Their task involved unfamiliar faces. The results showed that when the target face had served as the distractor during the previous trial, responses were slower, indicating that the distractor was inhibited (an effect referred to as negative priming). This seems to indicate that distractors depicting faces are subjected to inhibition; however, as noted by the authors, external features (especially hair) were not removed from the faces and thus the negative priming may reflect inhibitory processing of non-facial features. A similar argument can be made regarding the evidence of inhibition of previously cued unfamiliar faces [24], [25]. In addition, it may be the case that unfamiliar faces are subjected to more inhibition during selective attention than famous faces. Consistent with this possibility, Gazzaley et al. [26] reported evidence of inhibitory processing of unfamiliar distractor faces.

One seemingly odd aspect of our results is that the positive compatibility effect elicited by upright distractor faces was no more robust than that elicited by inverted distractor faces. Given that faces are particularly demanding of attention, one might have expected upright distractor faces to trigger stronger compatibility effects, especially given the famous status of the faces. However, considering that faces uniquely suffer from stimulus-specific capacity limits such that attending to a face can exhaust resources and limit processing of additional faces [27], [28], we suggest that face-specific capacity limits attenuated the influence of upright distractor faces, resulting in positive compatibility effects of similar magnitudes for upright and inverted faces.

The article "Famous Faces Demand Attention Due to Reduced Inhibitory Processing" was published in 2011. Journal: PLoS One.

A limitation of the current study is that the degree of familiarity was not matched across the stimuli used as non-face objects and upright faces; thus, we cannot rule out the possibility that the reduced inhibitory processing reported here for upright faces reflects the familiarity of the stimuli rather than engagement of face processing. However, it is worth noting that the stimuli used as non-face objects were familiar (the images depicted a butterfly and a wheel). Furthermore, negative compatibility effects occurred when consonants served as the stimuli (manuscript under review). Together, these experiments with familiar non-face stimuli suggest that familiarity does not prevent negative compatibility effects from mounting.

### Distractor inhibition during selective attention

Our data revealed that the contribution of distractor inhibition to focused attention depended on whether the distractor engaged face processing. This result provides novel evidence that the use of inhibition during selective attention is stimulus specific, which highlights the flexibility of inhibitory processing during focused attention. Importantly, this result also sheds new light on previous suggestions that distractor inhibition does not contribute to our ability to selectively attend, given that the supporting evidence came from a task that used famous faces as distractors [17], [29]. Egner and Hirsch [17] measured activation of the face-sensitive brain region (fusiform face area, FFA) while participants categorized names that appeared superimposed on a distractor face portraying a famous actor or politician. The results showed that FFA activity was not suppressed, which led to the suggestion that inhibition does not contribute to selective attention. Given the unique resilience of faces to selective attention (evidenced in these authors' data by a 41 ms compatibility effect for face distractors versus a 14 ms compatibility effect for name distractors), we suggest that the absence of evidence of inhibition may be specific to face distractors. Moreover, we recommend that future studies investigating mechanisms of selective attention avoid using face stimuli unless face processing is the specific topic of investigation.

### Conclusions

The current research provides novel evidence that distractors that portray faces are subject to less inhibitory processing, and this reduced inhibition could contribute to the difficulty people experience ignoring faces. Future research is required to determine whether reduced inhibitory processing is specific to famous faces, or whether faces in general are subjected to less inhibitory processing regardless of the status of the person portrayed.
